The article "Deformation Adjustment with Single Real Signature Image for Biometric Verification Using CNN" was retracted in 2023. Reasons: signs of a paper mill; compromised peer review; unreliable results or conclusions.

# Deformation Adjustment with Single Real Signature Image for Biometric Verification Using CNN

**DOI:** 10.1155/2022/4406101

**Published:** 2022-06-25

**Authors:** Rakesh Kumar, Mala Saraswat, Danish Ather, Muhammad Nasir Mumtaz Bhutta, Shakila Basheer, R. N. Thakur

**Affiliations:** ^1^Department of Computer Engineering & Applications, GLA University Mathura, Mathura-281406, India; ^2^Department of Computer Science and Engineering, ABES Engineering College Ghaziabad, India; ^3^Department of Computer Science & Engineering, School of Engineering & Technology Sharda University, Grater Noida, India; ^4^Computer Science and Information Technology (CSIT), College of Engineering, Abu Dhabi University, P.O. Box 5991, Abu Dhabi, UAE; ^5^Department of Information Systems, College of Computer and Information Science, Princess Nourah Bint Abdulrahman University, P.O. Box 84428, Riyadh 11671, Saudi Arabia; ^6^LBEF Campus, Kathmandu, Nepal

## Abstract

Signature verification is the widely used biometric verification method for maintaining individual privacy. It is generally used in legal documents and in financial transactions. A vast range of research has been done so far to tackle different system issues, but there are various hot issues that remain unaddressed. The scale and orientation of the signatures are some issues to address, and the deformation of the signature within the genuine examples is the most critical for the verification system. The extent of this deformation is the basis for verifying a given sample as a genuine or forgery signature, but in the case of only a single signature sample for a class, the intra-class variation is not available for decision-making, making the task difficult. Besides this, most real-world signature verification repositories have only one genuine sample, and the verification system is abiding to verify the query signature with a single target sample. In this work, we utilize a two-phase system requiring only one target signature image to verify a query signature image. It takes care of the target signature's scaling, orientation, and spatial translation in the first phase. It creates a transformed signature image utilizing the affine transformation matrix predicted by a deep neural network. The second phase uses this transformed sample image and verifies the given sample as the target signature with the help of another deep neural network. The GPDS synthetic and MCYT datasets are used for the experimental analysis. The performance analysis of the proposed method is carried out on FAR, FRR, and AER measures. The proposed method obtained leading performance with 3.56 average error rate (AER) on GPDS synthetic, 4.15 AER on CEDAR, and 3.51 AER on MCYT-75 datasets.

## 1. Introduction

The biometric system utilizes an individual's physiological or behavioural characteristics for identification, verification, and authentication. The invariable physiological characteristics include DNA, iris, fingerprint, palm, and facial expression [1, 2], whereas behavioural traits cover voice, signature, and handwriting [1, 3, 4]. Physical characteristics such as fingerprint and iris are often used because of their high performance. However, handwriting signatures are still being used and researched due to their ubiquitous use and cultural acceptance for personal authentication. Over centuries, its presence in legal documents, property wills and testaments, agreements, contracts, administrative records, and other legal and financial documents established it as a valuable trait. In the past, manual signature verification systems have substantially been used, but they are time-consuming and error-prone. Hence, research has been carried out on automating the verification of handwritten signatures since the decade of 1970 [5]. It justified the research community's extensive investigation and needs industry efforts to develop better products on researched technologies.

Biometric signature systems are involved in two scenarios, namely identification and verification. In the case of signature identification, the task is to retrieve similar signature samples from a signature repository when a signature is provided as a graphical query. In comparison, the signature verification system decides whether the same signer produces a given query signature or not. Thus, the signature verification system is used to classify given handwritten signature samples as genuine or forgeries. The broad categories of forgeries are random, simple, and skilled. This categorization is based on the availability of the user's name and signature to the forger. In the first category, the forger does not have information about both the factors. Due to this reason, the forger presents a signature with a different shape and looks very different in a holistic view. In contrast, the forger knows the user's name in the category of simple forgery. Hence, the forger can produce a much similar signature compared with a genuine signature if a user uses his name or subpart of it as a signature, whereas in the case of skilled forgery, the forger possesses information about the user name and the signature. It helps the forger practice the genuine signature and produces an almost similar signature to the genuine one. Due to this reason, detecting the forged signature in the case of skilled forgery is challenging.

Depending on the signature acquisition method, signature verification systems are either online or offline [6, 7]. If the acquisition method stores the signature as a sequence of pen placement points over time, then the corresponding system is an online signature verification system. An example of such an acquisition device is digitizing tablets. Additional information is also available in digitizing tablets, such as pen's inclination and tip pressure. In contrast, the offline signature system relied on devices such as digital cameras, in which the signature is considered as an image [8]. This work is mainly focused on the offline signature verification system. The signature image has been considered a static representation of the signature for this work.

Offline signature verification can follow two different approaches namely writer-dependent and writer-independent [9]. In the writer-dependent signature verification system, a model has been trained with a genuine and forged signature for a particular writer. During inference, the model has to decide based on the similarity measure between the query signature and the genuine signature. In case, if verification is needed for a new writer, a separate model needs to get trained, which is the major drawback of writer-dependent signature verification. In comparison, the writer-independent signature verification method is a generic system and can be deployed for multiple writers. Thus, the writer-independent signature verification is more cost-efficient.

In the offline signature verification method, the feature representation is one of the most researched points by the researchers in the past [10]. For feature representation, many handcrafted features have been designed and effectively used in the case of handwritten signature verification [9, 11–21], [5, 21–31], 71, but after the advent of deep convolutional neural networks (CNNs), the manual engineering for the features is no more needed. It can be learned by the neural network with the help of provided data [12, 32–36]. The learned features rely on the training of CNNs to learn the representation of the signature image by minimizing the loss function during the training phase. These deep learning methods have achieved good performance, but still, they are facing some trivial issues in case of signature verification.

An important issue in the training of deep neural networks is the capability of discriminating two visually close signatures, especially in the case of skilled forgery. In the case of skilled forgery, two signatures holistically look similar but only suffer from local deformation, which makes the two signatures dissimilar. It motivates us to devise a novel semi-synthetic approach to add local deformation on the signature for generating the synthetic forged version of the original image. It helps to train the network, which works efficiently to handle the most difficult case of forgery in the case of signature verification.

Another fundamental issue is the data-hungry deep learning approaches. The deep learning methods need millions of images to get trained. Ideally, in the case of signature verification, a single genuine image should be present in the repository for verification with query signature image, but in most existing methods, a set of signatures has been taken from the user (original signer) to train the deep learning method. However, to get rid of this data need for signature verification, we have mixed the signature data with the handwritten data. We consider the handwritten word as a genuine signature by a writer and the same word by another writer as a forged signature. A generic training has been conducted for the combined signature and word data. It helps to override the need for the vast amount of signature data for the training of the deep learning model for signature verification. Hence, the proposed system is writer-independent, and no separate model has been needed for a particular writer.

The rest of the study is organized into five sections.  Section 2 discusses the work related to the proposed method. In Section 3, the proposed approach is described in detail. In Section 4, the experimental setup has been described. The results and analysis of the proposed work have been discussed in Section 5. The conclusions have been drawn in Section 6.

## 2. Related Work

In document analysis research, biometric authentication is referred as the unique identification of a person. This authentication can be categorized based on the behavioural and psychological traits of a person. Another categorization is soft (signature, keystrokes, voice and handwriting, gait, etc.) biometrics and hard (facial expression, fingerprint, palm print-based geometry, etc.) biometrics [37]. Soft biometrics refers to features that change frequently depending on the situation. On the other hand, hard biometrics includes most of the features that remain permanent until the particular features meet any serious accident. Signature verification and analysis is an important soft biometric feature for person authentication, which can vary in offline and online modes. From the psychological evidence, the signature habit of an individual is a motor plan encoded thought. The moment of the motor plane at any fixed moment of time produces a common trajectory. By considering the trajectory of signature as stable regions, Parziale et al. [38] presented a stability modulated based on dynamic time wrapping (SM-DTW) for dynamic signature verification and ensured that the dynamic signature verification is more suitable to detect forgery. DTW is used to compare the string of two signatures with time.

### 2.1. Online Signature Verification

Porwik et al. [39] used the swarm intelligence technique with the probabilistic neural network (PNN) for signature verification. The dynamic feature of signature is similarity coefficients, which are selected during the Hotelling reduction process. PSO is helpful to achieve the similarity coefficients from dynamic features of signature. In the signature verification process, PNN is optimized by PSO, which is nicely tuned to the data statics of PNN classifier. Dynamic signature verification can closely represent the behavioural biometrics, which can be viewed in signing moments and speaking. For solving the problem of dynamic signature verification, Zhang [40] proposed the combination of population-based algorithms and fuzzy set theory. The evaluation of the scheme is carried out with the ATVSSLT signature verification database. The research work by the authors is referred as a measure of globally changing features and later concluded that their scheme provides a satisfactory solution for the like dynamic signature verification. Zalasinski et al. [41] also presented the dynamic signature verification based on selecting the most main partition. The key features of dynamic signature may include the change in the pressure of holding the pen and speed at particular word from the initial to middle and middle to final end of the signature. The method is primarily focused on the partition of particular parts of the signatures. Therefore, the approach increases the precision of signature processing and adapts the specific signature by removing redundant information. Dynamic methods and fuzzy set theory are used for weighted part signatures, which is a novel contribution.

### 2.2. Offline Signature Verification

Zouari et al. [42] proposed the offline signature verification on the basis of the algebraic geometry of the signature. They used partial order sets of the grids arranged in the form of lattice. Okawa [43] proposed a novel method by the fusion of the Fisher vector and KAZE features for offline signature verification. KAZE features are better to provide background information and remove the noise. The use of PCA with FV reduces the dimensionality issues and provides security by hiding the original signature. Sharif et al. [44] proposed the offline signature verification using very basic methods of feature extraction and feature processing. Initially, from the signature images binary map is prepared, which is further divided into 16 sub-blocks. By applying GA, at the individual block of signature, the received features were classified with SVM. In [45], fuzzy similarity measure and symbolic representation techniques are used for the offline signature verification. Inter-valued symbolic data are created from LBP features of signature images and bitmap images. In general, signature duplication methods can be considered as an initiative towards the improvements in automatic signature verification. Duplicate dynamic signature generation methods include several state-of-the-art methods such as kinematic model of motor system regarding neuroscience, nonlinear distortion, and affine transformation [46]. Research on static signature duplication is limited to achieve the recent advancements in human behaviour modelling. Diaz et al. [47] firstly proposed cognitive duplication of signature behaviour algorithm to develop an offline duplicate signature generation system. During the signing process, spatial cognitive maps of human behaviour and motor system were generated with the help of linear and nonlinear transformations.

Deep convolution neural networks have immensely justified its performance in image classification, natural language processing, and several social media analytics [48]. The toughest challenge in offline signature verification is the absence of dynamic features, which can be easily helpful to catch the skill forgery. Hafemann et al. [49] presented broad literature on the problem of offline signature verification and concluded that handcrafted feature extraction methods are super shaded by deep learning. They further added better fusion of features, augmentation of datasets, and important analysis of ensemble learning and deep learning. For keeping good features that maintain the system performance, Hafemann et al. [49] proposed learning from signature images with writer-independent mode using CNN. In the experiments, the training sample and generalization samples are kept separate. Hafemann et al. [49] presented a fixed-size representation scheme for offline handwritten signature verification of different sizes. From evolution in deep learning, it is ensured that handcrafted features have been down-shaded by the features automatically extracted from the deeply stacked layers in neural network. By utilizing pyramidal pooling, Hafemann et al. [49] added fixed-size input to network layers during varied range signatures from individual users.

From the literature, it has been found that the dynamic signature verification is more efficient than offline signature verification and a widely accepted person's authentication method, but the issues with dynamic signature verification are plenty of samples required to maintain the performance. For mitigating the issues, Daiz et al. [47] proposed signature verification with only single reference. Inspired from [47], in this work, we also introduced the method, which only needs a single reference image in the offline signature verification method.

## 3. Proposed Work

The overall workflow of the proposed signature verification system is depicted in Figure 1. The system has a preprocessing phase followed by an affine alignment of given query signature images. After the affine alignment of the query image with a reference image, local features are extracted from both images. Further, the features from the reference signature are matched with their neighbourhood feature in the query image and a similarity score is calculated. The signature verification decision is taken based on this similarity score.

### 3.1. Conceptual Background

The basic building block of deep learning frameworks originated from the black-box architecture of deep neural network. A brief idea of the components used for developing the deep neural network model for biometric verification system is mandatory to present in the following subsections.

#### 3.1.1. Convolution Neural Layer

The deep convolutional neural network is multilayered neural network and is recently used in various challenging problems [50–52]. The neurons of a convolution layer are connected to the local section of the input data. The receptive field of a neuron is the extent of its scope in input data, and it is increased by stacking the convolution layers. The convolution operation is given as equation (1), where *CB*^*k*^ is the *k*^*th*^ convolution kernel weights and its bias term, respectively, and is expressing the convolution method.

(1) $$\begin{array}{c} {\text{OpMap}}_{k}=\left({\text{InMapCK}}_{k}\right)+CB_{k}. \end{array}$$

The operation of convolution is constructed by one or more combination of such kernels. All convolution layers are followed by batch normalization layer and leaky ReLU as activation function in the proposed model.

#### 3.1.2. Batch Normalization Layer

The work [53, 54] revealed that deep neural networks' training is complicated and has different hyperparameters. Generally, the computational graph of a deep neural model has higher depth, leading to the convergence problem. There are some techniques [53–57] suggested to fix this issue. The batch normalization (BN) layer [56] is used in the proposed model for handling convergence problem and accelerates the network's training. In general, the BN layer is applied just before the activation layer (refer to [56] for details).

#### 3.1.3. Activation Function Layer

The activation functions in a neural network work as the transfer functions. These layers transform the results of the previous layer to map it with the given ground truth. Two kinds of activation functions are the linear activation function and the nonlinear activation function. In deep neural networks, different nonlinear functions are employed as the activation. These functions are generally introduced to maintain nonlinearity concept in the network. We have adopted various classes of different activation functions as described in the following subsections.

*(1) Leaky ReLU*. It is a linear rectified function, which is in short recall as ReLU. The output of ReLU function is zero for negative input, and otherwise, input remains unchanged (refer to equation (2)). In back propagation [58], the model parameters are updated by nonnegative input values. This leads to the dying ReLU problem; therefore, the leaky ReLU activation function is applied in our network to address this issue. Here, the negative slope *α* is not zeros but has a small value, which creates its derivative nonzeros for any input data (*α*=0.01 in our experiments). The function corresponding to mathematical representation is given by equation (2), and its derivatives are given by equation (3). The corresponding functions are also depicted in Figure 2.

(2) $$\begin{array}{c} \text{ReLU}\left(z\right)=\text{max}\left\{z,0\right\}, \end{array}$$

(3) $$\begin{array}{c} f\left(z\right)=\left\{\begin{array}{c} \alpha z,z<0. \end{array}\right. \end{array}$$

*(2) Hyperbolic Tangent Activation Function*. It is a kind of logistic sigmoid activation function, which has the important interpretation of the biological neurons. The main characteristic of hyperbolic tangent (tanh) function is having higher derivatives vanishing near zero. This is because the hyperbolic tangent function maintains its suitable property to learn the discriminative features from a higher class of varied data samples. The range of the tanh function is in the range of [−1,1]. The tanh function and its derivatives are dispensed in Figure 2 and obtained by equations (4) and (5), respectively. This activation function incorporates the recurrent network units (GRU and LSTM).

(4) $$\begin{array}{c} \text{tanh}z=\frac{e^{z}-e^{-z}}{e^{z}+e^{-z}}, \end{array}$$

(5) $$\begin{array}{c} \text{tanh}\prime z=1-{\text{tanh}}^{2}z. \end{array}$$

*(3) Sigmoid Activation Function*. The property of sigmoid activation function yields its normalized score in the range of [0,1] at the output scale. The mathematical expression of sigmoid function and its derivatives are explained in the figure below and calculated using equations (6) and (7), respectively. GRU and LTM unit present in recurrent network utilize the activation function for computing the corresponding activation values.

(6) $$\begin{array}{c} \sigma \left(z\right)=\frac{1}{1+e^{z}}, \end{array}$$

(7) $$\begin{array}{c} \sigma \prime \left(z\right)=1-\sigma \left(z\right). \end{array}$$

#### 3.1.4. MaxPool Layer

The MaxPool layer [59] is used to increase the receptive field of the network. This operation reduces (spatial dimensions) the size of the feature maps and decreases the computation cost. The reduction is applied only to the height and width of input data. The number of feature channels remains unchanged. It is similar to the sliding window approach with the selection of maximum element operation. The reduction in the size depends on the stride of the sliding operation. The proposed network utilizes a pooling size 2 × 2 and strides 2 × 2 for the pooling operation. The pooling is a nonparametric layer; therefore, there are no parameters for learning.

### 3.2. Preprocessing

A preprocessing step is not a vital phase for a convolutional neural network-based system, but it can reduce the total training time and sometimes improve the performance of the system. Besides this, it is also instrumental in representing the input data appropriately for the subsequent phases of the system. In this work, we are incorporating greyscale conversion of colour images and their intensity normalization as prepossessing steps. After converting a colour image into a greyscale image, it is resized such that its smaller side becomes 80 pixels. Besides this, we rotated the images such that the smaller side of the image becomes its height. Finally, its intensities are normalized such that the background pixels on the image became black or near to black, and the foreground pixels (signature pixels) became white or near to white (refer to Figure 3). Here, we are not converting the signature image into black and white; instead, it is still grayscale, but the background is black as we are using it as the padding in other sections of the system.

### 3.3. Affine Alignment

To understand the importance of this phase, let us assume that we have two different signature images of the same signer and try to find out their differences. There are two types of differences between these images: (1) global difference and (2) local difference. The global difference is caused by the shift in the position of signature, size, and shape variance and the orientation of its principal axis, whereas the local difference is caused by the deformation of each pixel in the form of its position displacement and colour intensity changes (refer to Figure 4).

In this phase, the proposed system analyzes the global differences by predicting the affine transformation of query signature image with respect to reference signature image. To predict the affine transformation of query image, the proposed system utilizes two trainable neural networks: (1) CNN-1 : convolution neural network and (2) FFNN-1 : feed-forward neural network. The overview of this phase is depicted in Figure 4 with the CNN-1 and FFNN-1 architecture.

Here, first of all the query and reference signature image are processed with CNN-1. This network produced 14*∗*64-dimensional vector for each image. These vectors (query image and reference image) are concatenated and passed to the FFNN-1. The FFNN-1 yields different parameters of affine transformation matrix. The architectural and parametric design detail of CNN-1 is given in Figure 4 and Table 1. Similarly, for FFNN-1 they are shown in Figure 4 and Table 2. The training procedure of this affine alignment network is explained in Subsection 3.4.

### 3.4. Training of Affine Alignment Network with Semi-Synthetic Dataset

The training of this network section is also a challenging task as we do not have labelled dataset having the affine transformation variation with ground truth. Therefore, we decided to go for a semi-synthetic dataset. Here, we collected signature images from all the datasets under consideration (refer to subsection 4.1) and handwritten word image samples from various datasets such as IAM [60] and CVL [61]. Considering these image samples as reference image, we applied a random affine transformation to generate query images. We utilized the random rotation with rotation angle *θ*_rotation_ ∈ [−45,45], random shearing with shearing angle *θ*_shearing_ ∈ [−20,20], and random scale *S*_*x*_, *S*_*y*_ ∈ [0.5, 2.0] for random affine transformation (all the transformations are with respect to the center of the image). In this way, we have collected a pair of reference and query image with their corresponding transformation parameters. Utilizing this information, we have trained the affine alignment network.

A affine transformation matrix is defined by equation (8). In our case, it is the combination of different elementary transformations such as translation, scale, shear, and rotation. The transformation matrix corresponding to these elementary transformations is given by equation (9).

(8) $$\begin{array}{c} \text{AffineTransformation}=\left[\begin{array}{ccc} b_{1} & c_{1}\\ a_{2} & b_{2} & c_{2}\\ 0 & 0 & 1 \end{array}\right], \end{array}$$

(9) $$\begin{array}{c} \text{Translation}=\left[\begin{array}{ccc} 0 & t_{x}\\ 0 & 1 & t_{y}\\ 0 & 0 & 1 \end{array}\right],\;\\ \text{Shear}=\left[\begin{array}{ccc} sr_{x} & 0\\ sr_{y} & 1 & 0\\ 0 & 0 & 1 \end{array}\right],\;\\ \text{Rotation}=\left[\begin{array}{ccc} -\sin\theta & 0\\ \sin\theta & \cos\theta & 0\\ 0 & 0 & 1 \end{array}\right]. \end{array}$$

### 3.5. Local Feature Extraction and Matching

Once the query image and reference image are aligned by transforming the reference image as affine transformation parameter (or transforming the query image as inverse affine transformation), we acquire the local features in both signature images. The local features are acquired by processing these images from the CNN-2. This network is a convolutional neural network, its architecture is depicted in Figure 5, and layered description is given in Table 3.

### 3.6. Local Feature Matching

This phase is responsible to handle the local differences in query image and reference image. The feature map (output of a CNN) generated by CNN-2 represents the neighbourhood region of size 44 × 44 pixels of a cell size 4 × 4 pixels. This representation is a 64-dimensional vector for each cell in feature map. Although the affine alignment phase already tackles major alignment issues, the pixel displacement can cause the local misalignment. Therefore, we calculate the Euclidean distance of a cell region in reference image with its 9 corresponding neighbours (3 × 3 window proximity) in the query image. The neighbouring cell in query image having the lowest distance is selected as the match for the corresponding cell in reference image.

### 3.7. Signature Verification Decision

This is the final step in the proposed signature verification system. Here, the matching distance of a cell in reference images is used in making a decision. It is possible that a genuine signature has some portion of signature extra or lesser with respect to reference signature (generally length of underline). So, here we need two levels of decision. First, we calculate the ratio (we call it *DMR*: distance matching ratio) of number of cells that have lesser matching distance than a predefined threshold (*Th*_*MD*_) with respect to number of cells that have it higher. We can further analyze a signature if it has *DMR* higher than a predefined threshold (*Th*_*DMR*_). The selection of *Th*_*DMR*_ depends upon the extent of extra signature that is allowed. In the proposed work, we have selected it as 4 (80% of total cell should be lower than *Th*_*MD*_). If a query signature gets *DMR* lesser than *Th*_*DMR*_ (in our case 4), then we simply discard the query signature. If the query signature passes the *Th*_*DMR*_, then we calculate its similarity score with respect to reference signature.

The similarity score is the mean of matching distance of all cell regions, which has matching distance lesser than *Th*_*MD*_.

## 4. Experimental Setup

### 4.1. Datasets

MYCT—this is offline signature verification dataset consisting of 75 writers. The name of the dataset is referenced from the project on science and technology under the Ministry of Spanish (Ministerio de Ciencia y Tecnologı'a) [62]. The dataset was prepared from 15 simple signatures and 15 simulated signatures along with corresponding figure prints. The resolution of all images of signatures was maintained at 600 dpi. The dataset is useful to develop the biometric algorithms in several secured domains. GPDS—this is an offline signature verification database developed in signal processing laboratory (Grupo de Procesado Digital de la señal) GPDS at University of Las Palmas de Gran Canaria, Spain [63]. GPDS consists of 24 genuine signatures and 30 forgery signatures from each of 960 individuals. The signatures are black and white format with 300 dpi. During the collection of samples, two different sizes of boxes are chosen, one is 5 cm by 1.8 cm and another is 4.5 cm by 2.5 cm. CEDAR—this is an online handwritten text database consisting of the samples of handwritten text of tablet and line of text collected from 200 writers [64]. CEDAR signature recognition dataset was developed at Buffalo University. The dataset consists of 24 samples for each genuine and simulated signature from 55 enrolled forgeries. The simulated signatures include both simple and forgeries. The dataset is very large as it contains 105,573 numbers of words.

### 4.2. Evaluation Criteria

The results obtained from the proposed work are compared with current state-of-the-art methods on different standard datasets and with different evaluation criteria. We have tested the performance of the system through writer-independent signature verification task considering all reference signatures as a separate entity. We are listing the performance of the proposed system with three evaluation measures such as (1) FRR, (2) FAR, and (3) AER.

#### 4.2.1. FRR

It stands for false rejection rate, a very important evaluation parameter in the biometric system to measure the likelihood that the biometric-based security system incorrectly rejects the access attempt made by the authentic user of the system. Mathematically (equation (10)), FRR is calculated as a ratio of the total counts of false rejections and total identification attempts.

(10) $$\begin{array}{c} \text{FRR}=\frac{FN}{TP+FN}. \end{array}$$

#### 4.2.2. FAR

False acceptance rate or FAR is also a likelihood measure to determine that the biometric system incorrectly accepts the access attempt by the unauthentic user. In terms of mathematical formula, FAR (equation (11)) of a biometric system is the ratio of total counts of false acceptances and total number of identification attempts.

(11) $$\begin{array}{c} \text{FAR}=\frac{FP}{FP+TN}. \end{array}$$

#### 4.2.3. AER

The average error rate or AER is termed as the best threshold value at which the curve of FAR and FRR meets at a point. It generally determines the stability of the system. It is mathematically computed as an average of FRR and FAR as follows:

(12) $$\begin{array}{c} \text{AER}=\frac{FAR+FRR}{2}. \end{array}$$

## 5. Results and Analysis

The proposed system has been extensively validated on the three public datasets of signature verification, namely MCYT-75, CEDAR, and GPDS. The proposed method is also compared with other state-of-the-art methods. The evaluation results for the MCYT-75 dataset are summarized in Table 4. From Table 4, it has been observed that for the 5G and 12G training samples, our proposed method has reported the least average error rate. The proposed system has achieved the least false acceptance rate (FAR) and false reject rate for 5G, 10G, and 12G training samples. This shows the proposed approach's robustness compared with other state-of-the-art methods for the MCYT-75 dataset.

For the CEDAR dataset, the quantitative results, along with the state-of-the-art approaches, are mentioned in Table 5. From Table 5, it has been found that for independent writer setting, our method is best performing as compared to the other 12G training samples. Even the proposed method has achieved the least average error rate for 12G compared with all methods (writer-independent and writer-dependent). The proposed system also achieves least false rejection rate and false acceptance rate for all settings of training samples.  Figure 6 presents the average error rate (AER) for different samples taken from all three mentioned datasets. It also presents the comparative results against the mentioned state of the art. Another set of comparisons is shown in Figure 7 against the different training samples of independent and dependent writers with their rate of performance.

The impact of the proposed method for the GPDS synthetic dataset is summarized in Table 6. The proposed method has achieved the best results on the AER metric for all training sample settings. The proposed method has also outperformed [44] on the metric of false rejection rate. From Tables 4–6, it is observed that the robustness of the proposed approach is compared with other existing approaches and has been validated with satisfactory measures.

## 6. Conclusion

Generally, signatures are composed of multiple components, and most of them do not provide the necessary information. For example, the date and curved line used below the signature must be ignored since it does not add any information for writer identification. Alternatively, this may help to remove the processing overheads. Interpersonal similarity and high intrapersonal variability are the challenging factors for achieving satisfactory performance to generalize offline signature verification. This may be supposed to extract the most discriminant and stable feature sets from the wide variety of geographical-invariant signers. In this study, we presented a practical verification problem against the forgeries. In the context of feature extraction for writer-independent signature verification, the line-up future directions may be planned to fuse nonhandcrafted features. In the case of adversarial machine learning in the security domain, an interesting future direction can be added to analyze the impact of sharp physical attacks by printing the adversarial noise over the signatures. According to the writer's perspective, another future line can be encouraged to develop a better deep network than the Siamese network and the loss functions to introduce versatile reference signatures. Signature localization is also an important domain that can assist in signature verification in an image.

## Figures and Tables

**Figure 1:** Overall workflow of proposed signature identification and verification (SIV) system.

**Figure 2:** Different activation functions.

**Figure 3:** Left figure (a) shows the preprocessing steps used in the proposed system. Figure (b) in the right side is exemplifying the global deformation in pair of target signature images.

**Figure 4:** Affine alignment of query signature image with reference signature image.

**Figure 5:** Local feature extraction and matching.

**Figure 6:** Comparison of AER on MYCT-75 (a) CEDAR (b) and GPDS (c) datasets along with different sizes of data samples.

**Figure 7:** Overall comparative performance in terms of FRR, FAR, and AER on *MYCT* − 75, GPDS, and CEDAR datasets.

**Table 1:** Architecture description of the CNN-1: convolutional neural network-1 section of the proposed system.

Layer	#Kernel	Kernel size	#Parameter	Output size
Input	0	0	0	*H* × *W* × 1
*C*_1_^1^	32	5 × 5	832	*H* × *W* × 32
*C*_1_^2^	32	3 × 3	9248	*H* × *W* × 32
*C*_2_^1^	64	3 × 3	18496	*H*/2 × *W*/2 × 64
*C*_2_^2^	48	3 × 3	27696	*H*/2 × *W*/2 × 48
*C*_2_^3^	64	3 × 3	27712	*H*/2 × *W*/2 × 64
*C*_3_^1^	128	3 × 3	73856	*H*/4 × *W*/4 × 128
*C*_3_^2^	64	3 × 3	73792	*H*/4 × *W*/4 × 64
*C*_3_^3^	128	3 × 3	73856	*H*/4 × *W*/4 × 128
*C*_4_^1^	64	3 × 3	73792	*H*/8 × *W*/8 × 128
Total number of parameters in CNN-1: 379280				

**Table 2:** Architecture description of the FFNN-1: feed-forward neural network-1 section of the proposed system.

Layer	#Neurons	#Parameter	Output size
Input	0	0	128
*D*_*t*_^1^	64	8256	64
*D*_*t*_^2^	128	8320	128
*D*_*t*_^3^	64	8256	64
*D*_*t*_^4^	2	130	2
*D*_*r*_^1^	64	8256	64
*D*_*r*_^2^	128	8320	128
*D*_*r*_^3^	64	8256	64
*D*_*r*_^4^	2	130	2
*D*_*s*_^1^	64	8256	64
*D*_*s*_^2^	128	8320	128
*D*_*s*_^3^	64	8256	64
*D*_*s*_^4^	2	130	2
Total number of parameters in FFNN-1: 74886			

**Table 3:** Architecture description of the CNN-2 : convolutional neural network-1 section of the proposed system.

Layer	#Kernel	Kernel size	#Parameter	Output size
Input	0	0	0	*H* × *W* × 1
*C*_1_^1^	32	3 × 3	320	*H* × *W* × 32
*C*_1_^2^	32	3 × 3	9248	*H* × *W* × 32
*C*_2_^1^	32	3 × 3	18496	*H*/2 × *W*/2 × 32
*C*_2_^2^	48	3 × 3	27696	*H*/2 × *W*/2 × 48
*C*_2_^3^	32	3 × 3	27712	*H*/2 × *W*/2 × 32
*C*_3_^1^	64	3 × 3	73856	*H*/4 × *W*/4 × 64
*C*_3_^2^	48	3 × 3	73792	*H*/4 × *W*/4 × 48
*C*_3_^3^	64	3 × 3	36928	*H*/4 × *W*/4 × 64
Total number of parameters in CNN-2: **268048**				

**Table 4:** Comparison of the proposed system with other (including current state-of-the-art) methods with MCYT-75 dataset.

Author	Verification type	No. of training sample	FRR	FAR	AER
[4]	WD	5G	32.4	26.84	—
		10G	22.93	22.04	—
[65]	—		6.67	12.44	9.56
[66]	WD	5G	23.25	4.53	—
		10G	12.61	7.53	—
[42]	WD	5G	4.48	25.19	5.62
		10G	4.96	17.21	3.45
[67]	WD	10G	12.53	13.16	—
		5G	15.47	13.42	—
[44]	WD	5G	6.67	6.67	6.67
		10G	6.25	5.67	5.96
		12G	3.67	6.67	5.0
Ours	WI	5G	4.12	4.48	4.30
		10G	3.68	3.96	3.82
		12G	3.49	3.53	3.51

**Table 5:** Comparison of the proposed system with other (including current state-of-the-art) methods with CEDAR dataset.

Author	Verification type	No. of training sample	FRR	FAR	AER
[68]	WI	24G	—	—	8.33
[69]	WD	16G	6.36	5.68	6.02
[33]	WD	12G	9.36	7.84	8.60
[42]	WD	5G	4.44	15.91	3.64
		10G	5.83	11.52	2.74
[70]	WI	4G	—	—	8.70
		8G	7.41	8.25	7.83
		12G	—	—	5.60
[44]	WD	5G	12.5	8.33	10.41
		10G	8.33	4.17	6.25
		12G	4.67	4.67	4.67
Ours	WI	5G	4.32	7.84	6.08
		10G	5.72	4.12	5.92
		12G	3.97	4.33	4.15

**Table 6:** Comparison of the proposed system with other (including current state-of-the-art) methods with GPDS synthetic dataset.

Author	Verification type	No. of training sample	FRR	FAR	AER
[67]	WD	10G	5.80	29.49	—

[44]	WD	5G	8.33	10	9.16
		10G	12.5	3.33	7.92
		12G	6.67	4.16	5.42
		16G	4.16	3.33	3.75

Ours	WI	5G	6.12	7.68	6.90
		10G	5.96	6.32	6.14
		12G	4.84	4.46	4.65
		16G	3.65	3.47	3.56

## Data Availability

The data used to support the study are cited within the article and are publicly available.
